# *Evodiae fructus* Extract Inhibits Interleukin-1*β*-Induced MMP-1, MMP-3, and Inflammatory Cytokine Expression by Suppressing the Activation of MAPK and STAT-3 in Human Gingival Fibroblasts In Vitro

**DOI:** 10.1155/2021/5858393

**Published:** 2021-08-31

**Authors:** Hyun-Kyung Song, Eun-Mi Noh, Jeong-Mi Kim, Yong-Ouk You, Kang-Beom Kwon, Young-Rae Lee

**Affiliations:** ^1^Herbal Medicine Research Division, Korea Institute of Oriental Medicine, Yuseong-daero 1672, Yuseong-gu, Daejeon 34054, Republic of Korea; ^2^Department of Oral Biochemistry and Institute of Biomaterials, Implant School of Dentistry, Wonkwang University, Iksan City, Jeonbuk, Jeollabuk-do 570-749, Republic of Korea; ^3^Department of Biochemistry, Institute of Medical Science, Chonbuk National University Medical School, Jeonju, Jeollabuk-do 560-182, Republic of Korea; ^4^Department of Korean Physiology, Wonkwang University School of Korean Medicine, Iksan City, Jeonbuk, Jeollabuk-do 570-749, Republic of Korea

## Abstract

Periodontitis is a Gram-negative bacterial infectious disease. Numerous inflammatory cytokines, including interleukin-1*β* (IL-1*β*), regulate periodontitis pathophysiology and cause periodontal tissue destruction. In human gingival fibroblasts (HGFs), IL-1*β* stimulates the production of matrix metalloproteinases (MMPs) and proinflammatory cytokines via various mechanisms. Several transcription factors, such as signal transducer and activator of transcription 3 (STAT-3), activator protein 1 (AP-1), and nuclear factor-*κ*B (NF-*κ*B), regulate gene expression. Mitogen-activated protein kinases (MAPKs) regulate these transcription factors. However, the MAPK/STAT-3 activation signal in HGFs is unknown. We investigated the potential inhibitory effects of the extract of *Evodiae fructus* (EFE), the dried, ripe fruit of *Evodia rutaecarpa*, on MMP and proinflammatory cytokine expression in IL-1*β*-stimulated HGFs. EFE inhibited the expression of MMP-1, MMP-3, and proinflammatory cytokines (TNF-*α*, IL-6, and IL-8) in IL-1*β*-stimulated HGFs through the inhibition of IL-1*β*-induced MAPK/STAT-3 activation. Also, these results suggest that the EFE may be a useful for the bioactive material for oral care.

## 1. Introduction

Periodontitis is a serious inflammatory disease of the gums. It is most commonly caused by periodontal Gram-negative bacterial infections such as *Porphyromonas gingivalis* infection, causes connective tissue destruction and bone resorption around the teeth, and is the leading cause of tooth loss [1, 2]. *P. gingivalis* produces lipopolysaccharide (LPS), which is a major virulence factor, to induce inflammation [3]. LPS induces the expression of proinflammatory cytokines and inflammatory mediators, such as tumor necrosis factor-*α* (TNF-*α*), interleukin-1 (IL-1), IL-6, IL-8, E-prostaglandins (PGEs), and nitric oxide (NO) [4]. Among these, IL-1 plays a major role in periodontal tissue destruction by enhancing the expression of collagenic enzymes, including matrix metalloproteinases (MMPs) [5, 6].

Gingival connective tissue mainly consists of stromal cells, such as fibroblasts, and extracellular matrix (ECM). ECM is a complex structure of mucopolysaccharides and fibrin, including collagens, elastin, fibronectin, glycosaminoglycans, and laminins, which structurally supports the cells and mechanical strength of tissues [7, 8]. MMPs are a family of structurally related ECM-degrading enzymes and are associated with several destructive processes, including inflammation, tumor invasion, and periodontitis [9, 10]. Inflamed periodontal tissue, including epithelial cells and fibroblasts, expresses various types of MMPs [11]. Especially, gingival fibroblasts are known to produce MMP-1, -2, -3, -7, -8, -9, and -13 and to be involved in periodontal tissue destruction [12–14]. MMP-1 (collagenase I) and MMP-3 (stromelysin) play important roles in periodontal diseases [6, 12, 15]. MMP-1 mainly degrades the collagen present in periodontal tissues during periodontal disease progression [16]. MMP-3 disassembles ECM structural substances and induces the release of some proenzymatic MMP forms [16–18]. Human gingival fibroblasts (HGFs) are known to secrete MMP-1 and MMP-3 in response to stimulation with IL-1 [6, 19, 20].

IL-1 is an important and multifunctional cytokine associated with host immune and inflammatory reactions [21]. Previous studies have suggested the importance of IL-1 in the development of periodontal diseases [15, 22, 23]. Through its various biological activities, IL-1 induces a variety of inflammatory reactions, including the synthesis of NO and reactive oxygen species (ROS) and the expression of PGEs, MMPs, and inflammation-related cytokines [24]. In addition, it is one of the most powerful inducers of MMPs in HGFs [25]. IL-1 activates MMP expression-related signaling pathways, including mitogen-activated protein kinase (MAPK), and transcription factors, such as signal transducer and activator of transcription 3 (STAT-3), activator protein 1 (AP-1), and nuclear factor-*κ*B (NF-*κ*B) [26–28]. In HGFs, IL-1*β* induces TNF-*α*, IL-6, IL-8, and MMP expression via the MAPK/NF-*κ*B/AP-1 signaling axis [20] and causes STAT-3 phosphorylation [29].

*Evodiae fructus* (EF) is the dried, ripe fruit of *Evodia rutaecarpa*, which has been used as an analgesic, antidiarrheal, antiemetic, and anti-inflammatory drug in Chinese traditional medicine [30, 31]. Alkaloids are the main active ingredients of EF, and recent studies have investigated the pharmacological activities of alkaloids such as evodiamine, hydroxyevocarpine, hydroxyevodiamine, evocarpine, isoevodiamine, higenamine, and rutaecarpine [31]. Especially, EF exerts anti-inflammatory effects by inhibiting proinflammatory cytokine production, ROS generation, and MAPK activation [32]. However, the anti-inflammatory effects of EF on HGFs have not yet been investigated.

Therefore, the hypothesis of the present study was that EFE could inhibit inflammatory reactions in IL-1*β*-stimulated HGFs. In this study, we investigated the effects of the EF extract (EFE) on IL-1*β*-induced proinflammatory cytokine and MMP expression in HGFs. Furthermore, we demonstrated the signal pathways of anti-inflammatory effects of the EFE by detecting several inflammatory mediators such as MAPK, NF-*κ*B, AP-1, and STAT-3.

## 2. Materials and Methods

### 2.1. HGF Culture

HGFs were obtained from Lifeline Cell Technology (Walkersville, MD, USA). Cells were grown in Dulbecco's Modified Eagle's Medium (DMEM) supplemented with 10% heat-inactivated fetal bovine serum (FBS), penicillin 100 units/mL, streptomycin 100 *µ*g/mL, and Fungizone^®^ (amphotericin B) 0.25 *µ*g/mL at 37°C in a 5% CO_2_ atmosphere. Cells were passaged at a rate of one-third at regular intervals so that the monolayers did not exceed 70–80% confluence.

### 2.2. Reagents

EF water extract was purchased from the Korean Plant Extract Bank (CW02-075; Daejeon, Korea), and a 50 mg/ml stock was prepared in distilled water. Human MMP-1 and MMP-3 antibodies and recombinant human IL-1*β* were obtained from R&D Systems (Minneapolis, MN, USA). Anti-*β*-actin antibody, p38 inhibitor SB203580, JNK inhibitor SP600125, and ERK inhibitor PD98059 were purchased from Sigma-Aldrich (St. Louis, MO, USA). p-c-Jun antibody was purchased from Abcam (Cambridge, MA, USA). PCNA, p65, and p50 antibodies were purchased from Santa Cruz Biotechnology (Santa Cruz, CA, USA). p-STAT3, STAT-3, p-JNK, JNK, p-p38, p38, p-ERK, and ERK antibodies were obtained from Cell Signaling Technology (Beverly, MA, USA). High-glucose DMEM was purchased from HyClone (Logan, UT, USA). FBS and phosphate-buffered saline (PBS) were purchased from Gibco BRL (Gaithersburg, MD, USA).

### 2.3. Cell Viability Assay

The effect of the EFE on HGF viability was determined using the Cellrix^®^ Viability Assay Kit (Medifab, Seoul, Korea). Cells were seeded in each well of a 96-well plate and incubated for 24 h. EFE was added at various concentrations (0–100 *μ*g/ml), and the plate was further incubated for 24 h. Then, 10 *μ*l of assay reagent was added in each well, and the plate was incubated in the dark at 37°C for 1 h. After the incubation, the optical density at 450 nm was read on a microplate reader (Sunrise^™^, Tecan, Mannedorf, Switzerland).

### 2.4. Western Blot Analysis

HGFs were pretreated with 25 or 50 *μ*g/ml EFE for 1 h and then incubated with IL-1*β* at 37°C for 24 h. Collected cell pellets were lysed in radioimmunoprecipitation assay buffer (Thermo Fisher Scientific, Waltham, MA, USA) on ice. Total proteins were quantified using a BioSpec-nano instrument (Shimadzu, Kyoto, Japan). Proteins (25 *μ*g) were electrophoresed in a 10% sodium dodecyl sulfate-polyacrylamide gel at 100 V and transferred onto blotting membranes (GE Healthcare Life Sciences, Little Chalfont, UK). After blocking for 2 h, the membranes were incubated with primary antibodies diluted (1 : 1000) in blocking solution (5% skim milk or bovine serum albumin in TBS with Tween 20) at 4°C overnight and then with secondary antibodies for 1 h under gentle agitation. Protein bands were visualized using a Mini HD6 image analyzer (UVITEC, Cambridge, UK).

### 2.5. Enzyme-Linked Immunosorbent Assay (ELISA)

Cells were pretreated with the EFE for 1 h and then treated with IL-1*β* at 37°C for 24 h. Cell culture medium was collected after removing the particulates. MMP-1 and MMP-3 levels in the culture supernatants were determined using a Human Active MMP-1 Fluorokine E Kit and Human MMP-3 Quantikine ELISA Kit (R&D Systems, Minneapolis, MN, USA) according to the manufacturer's protocols.

### 2.6. Quantitative Reverse Transcription (RT-q) PCR

RNA was extracted from cultured cells using TRIzol® reagent (Invitrogen, Carlsbad, CA, USA). RNA concentrations were determined on the BioSpec-nano instrument. cDNA was synthesized from total mRNA (1 *μ*g) using the PrimeScript^™^ RT Reagent Kit (Takara, Shiga, Japan). mRNA levels of MMP-1, MMP-3, TNF-*α*, IL-6, IL-8, and glyceraldehyde 3-phosphate dehydrogenase (GAPDH) were determined by qPCR using SYBR^®^ Green reagent and a StepOnePlus Real-Time PCR System (both from Applied Biosystems, Foster City, CA, USA). Target mRNA levels were normalized to those of GAPDH as an internal control (Table 1).

### 2.7. Nuclear Fractionation

HGFs were prestimulated with EFE or MAPK inhibitors (SB203580, PD98059, and SP600125) for 1 h and then incubated with IL-1*β* for 3 h. Then, the cells were immediately washed twice with PBS. Nuclear proteins were isolated using NE-PER^®^ Nuclear and Cytoplasmic Extraction Reagents (Pierce Biotechnology, Rockford, IL, USA) per the manufacturer's protocol.

### 2.8. RNA Interference

Negative control small interfering RNA (siRNA) and STAT-3-specific siRNA were purchased from BIONEER (Daejeon, Korea). In brief, HGFs were transfected with 200 pmol siRNA using Lipofectamine RNAiMAX (Invitrogen, Carlsbad, CA, USA) according to the manufacturer's instructions in 60 mm dishes at 37°C for 48 h.

### 2.9. Statistical Analysis

All experiments were performed in triplicate. Statistical significance was evaluated using the analysis of variance (one-way ANOVA) followed by Tukey's multiple comparison test. *p* < 0.01 was considered significant.

## 3. Results

### 3.1. Effect of the EFE on IL-1*β*-Induced MMP-1 and MMP-3 Expression in HGFs

First, to evaluate the cytotoxicity of the EFE on HGFs, the cells were incubated with various concentrations of the EFE for 24 h. EFE treatment for 24 h did not significantly affect cell viability (Figure 1(a)). Thus, nontoxic concentrations (25 and 50 *μ*g/ml) of the EFE were used in subsequent experiments. To evaluate the effects of the EFE on IL-1*β*-induced MMP expression, MMP protein and mRNA levels were determined using western blotting and RT-qPCR, respectively. IL-1*β* significantly increased MMP-1 and MMP-3 protein expression, whereas the increases were significantly suppressed by the EFE (Figure 1(b)). Similarly, IL-1*β*-induced increases in mRNA levels were significantly suppressed by pretreatment with the EFE (Figures 1(c) and 1(d)). In addition, we evaluated the effects of the EFE on MMP-1 and MMP-3 secretion using ELISA, and IL-1*β*-induced MMP secretion was inhibited by the EFE (Figures 2(a) and 2(b)).

### 3.2. Effect of the EFE on IL-1*β*-Induced Proinflammatory Cytokine Expression in HGFs

To evaluate the effects of the EFE on proinflammatory cytokine expression in IL-1*β*-stimulated HGFs, cells were pretreated with 50 *μ*g/ml EFE for 1 h and then stimulated with IL-1*β* at 37°C for 0, 2, 4, 6, or 8 h. The mRNA levels of TNF-*α*, IL-6, and IL-8 were estimated by RT-qPCR. As shown in Figure 3, EFE suppressed the increases in TNF-*α*, IL-6, and IL-8 mRNA levels induced by IL-1*β* stimulation at several time points.

### 3.3. Effect of the EFE on IL-1*β*‐Induced MAPK/NF-*κ*B/AP-1 Activation in HGFs

To investigate the signaling pathway involved in EFE-mediated suppression of IL-1*β*-induced proinflammatory cytokine and MMP expression, we examined the effects of the EFE on the activation of MAPK and several transcriptional factors. In HGFs, MMP expression is regulated by the MAPK/NF-*κ*B or MAPK/AP-1 pathway [48]. Therefore, we confirmed that the EFE inhibited IL-1*β*-induced phosphorylation of MAPKs (p38, ERK, and JNK) (Figure 4(a)). To investigate the effects of the EFE on NF-*κ*B and AP-1 activation by IL-1*β*, we examined the nuclear translocation of p65, p50, and p-c-Jun by western blotting, which confirmed that the EFE did not affect IL-1*β*-induced activation of NF-*κ*B and AP-1 (Figure 4(b)). These results indicated that the EFE inhibits IL-1*β*-induced TNF-*α*, IL-6, IL-8, MMP-1, and MMP-3 expression through the inhibition of MAPK activation but does not involve the NF-*κ*B and AP-1 pathways in HGFs.

### 3.4. Effect of MAPK/STAT-3 Activation on IL-1*β*‐Induced MMP-1 and MMP-3 Expression

As the EFE did not inhibit either of the MAPK/NF-*κ*B and MAPK/AP-1 pathways and STAT-3 activation reportedly induced MMP expression and was affected by MAPK activation [33, 34], we investigated the potential association with STAT-3. As shown in Figure 5(a), IL-1*β* increased STAT-3 phosphorylation in the nuclear fraction of HGFs, which was inhibited by the EFE. To investigate whether MAPK signaling is directly involved in IL-1*β*-induced STAT-3 phosphorylation in HGFs, we evaluated the effects of MAPK inhibitors (p38: SB203580, ERK: PD98059, and JNK: SP600125) on IL-1*β*-induced activation of STAT-3 phosphorylation in HGFs. All three MAPK inhibitors inhibited STAT-3 phosphorylation at 3 h after IL-1*β* treatment (Figure 5(b)). Next, to investigate the association between STAT-3 and IL-1*β*-induced MMP-1 and MMP-3 expression, we knocked down STAT-3 expression using STAT-3 siRNA. STAT-3 knockdown reduced IL-1*β*-induced MMP-1 and MMP-3 protein expression (Figures 5(c) and 5(d)). This result indicated that IL-1*β*-induced MMP-1 and MMP-3 expression is regulated through MAPK/STAT-3 activation in HGFs.

## 4. Discussion

Periodontitis is the most prevalent inflammatory disease and is caused by periodontal Gram-negative bacterial infection [1]. Such infections induce an inflammatory reaction, leading to periodontal tissue destruction and bone resorption [35]. *P. gingivalis*, one of the most important bacteria in periodontal disease, produces LPS, a major toxin that induces inflammatory responses. LPS induces the production of various proinflammatory cytokines and mediators, such as IL-1, TNF-*α*, NO, and PGE2, in immune cells, which trigger the destruction of periodontal tissue by MMPs produced by gingival fibroblasts or inflammatory cells, including osteoclasts [11, 36]. MMPs play important roles in the degradation of the ECM and bone collagen matrix in periodontitis [37–39]. In active periodontitis, periodontal tissue loss and alveolar bone destruction are increased by MMPs and inflammatory cytokines [2, 38]. Various types of MMPs, including MMP-1, -2, -3, -8, -9, and -13, are involved in periodontal tissue destruction [12–14, 40]. Especially, MMP-1 and MMP-3 are important in periodontal diseases [12, 15, 41]. Therefore, unraveling the regulation of MMP-1 and MMP-3 may contribute to the development of treatments for periodontitis. Therefore, we investigated the potential inhibitory effects of the EFE on MMP-1 and MMP-3 expression in HGFs (Figures 1 and 2).

HGFs are a major cell type in periodontal tissue and secrete various inflammatory cytokines upon inflammatory stimuli, including bacteria and their pathogenicity factors [42–44]. IL-1 is an important proinflammatory cytokine present in inflammatory gingiva and plays essential roles in the pathogenesis of periodontitis [45, 46]. IL-1 is involved in the inflammatory response and ECM remodeling through the induction of various factors, including ROS, NO synthase, PGEs, cytokines, and MMPs [24]. Upon stimulation with IL-1*β*, HGFs produce TNF-*α*, IL-6, and IL-8 [47]. TNF-*α* is primarily secreted by immune cells such as fibroblasts and is a potent proinflammatory cytokine that induces the production of MMP, cytokines, PGE2, cell adhesion molecules, and molecules related to bone resorption [20, 48, 49]. IL-6 plays a crucial role in infected periodontal tissue as well as in bone resorption, osteoclast differentiation, and continuous tissue destruction [50]. IL-8 induces the migration of neutrophils to periodontal lesions, weakening periodontal tissue due to intracellular ROS production, MMP expression, and lysosomal enzyme release [51, 52]. This cytokine is highly expressed in periodontal tissue [53]. Our study findings suggest that the EFE may improve periodontal inflammation by inhibiting the expression of proinflammatory cytokines in HGFs (Figure 3).

IL-1*β* reportedly induces MAPK/NF-*κ*B and AP-1 signaling in HGFs [20, 54]. Furthermore, the MAPK/AP-1 and NF-*κ*B cascades mediate IL-1*β*-stimulated cytokine and MMP-1 expression in HGFs [20, 55]. To evaluate the mechanism underlying the inhibitory effect of the EFE on IL-1*β*-induced MMP and proinflammatory cytokine expression, we examined the effects of the EFE on MAPK/NF-*κ*B/AP-1 activation. EFE did not regulate MMPs through MAPK/NF-*κ*B/AP-1 activation (Figure 4). Therefore, we next investigated a potential association with STAT-3. It has been reported that intracellular, activated STAT-3 regulates the expression of MMPs and proinflammatory cytokines [33, 34, 56]. However, the association between STAT-3 and cytokine and MMP expression induced by IL-1 in HGFs had not been investigated. To evaluate the association between MAPK and STAT-3, we used inhibitors of p38 (SB203580), ERK (PD98059), and JNK (SP600125) and determined STAT-3 phosphorylation induced by IL-1*β*. While p-STAT-3 levels were increased in the IL-1*β*-treated group, the MAPK inhibitors were found to inhibit STAT-3 phosphorylation, suggesting an interaction between MAPK and STAT-3 (Figure 5(b)). Additionally, we confirmed that STAT-3 knockdown suppressed IL-1*β*-induced MMP-1 and MMP-3 expression (Figures 5(c) and 5(d)). These results are particularly relevant as this is the first report of MMP expression regulation by IL-1*β*-induced MAPK/STAT-3 activity in HGFs. Finally, we confirmed that the EFE inhibits IL-1*β*-induced STAT-3 phosphorylation (Figure 5(a)). However, since the EFE is an extract, not a single compound, further investigation is required to analyze the active compounds that exhibit the anti-inflammatory effects of the EFE. Additional studies will be necessary to confirm the anti-inflammatory effects of the EFE in periodontitis using an in vivo experimental model.

## 5. Conclusion

Taken together, this study demonstrated that the EFE inhibits IL-1*β*-induced MAPK/STAT-3 activation in HGFs and the expression of MMP-1 and MMP-3, which decompose various substrates present in periodontal tissue. The extract also inhibits several increased proinflammatory cytokines, such as TNF-*α*, IL-6, and IL-8. These results suggest that the EFE may be a useful bioactive material for oral care.

## Figures and Tables

**Figure 1:** Effect of the EFE on the viability of HGFs. Cells were seeded, incubated for 24 h, and treated with the EFE at 0, 6.25, 12.5, 25, 50, and 100 *μ*g/ml. Cytotoxicity of the EFE was investigated after treatment for 24 h (a). Cells were preincubated with 25 and 50 *μ*g/ml of the EFE for 1 h and then treated with IL-1*β* for 24 h. Western blot analysis was performed to determine MMP-1 and MMP-3 protein levels in HGF lysates (b). The MMP-1 and MMP-3 expression was analyzed using RT-qPCR (c, d). Data were presented as the mean ± SEM of three independent experiments. ^#^*p* < 0.01 vs. control; ^*∗*^*p* < 0.01 vs. IL-1*β*.

**Figure 2:** EFE inhibits IL-1*β*-induced MMP secretion. Cells were pretreated with the EFE for 1 h and then incubated with IL-1*β* for 24 h. Secreted MMP-1 (a) and MMP-3 (b) proteins were detected using ELISA. Data were presented as the mean ± SEM of three independent experiments. ^#^*p* < 0.01 vs. control; ^*∗*^*p* < 0.01 vs. IL-1*β*.

**Figure 3:** EFE inhibits IL-1*β*-induced proinflammatory cytokine mRNA expression in HGFs. HGFs were prestimulated with 50 *μ*g/ml of the EFE for 1 h and then incubated with IL-1*β* various times. Total cellular mRNA levels of TNF-*α* (a), IL-6 (b), and IL-8 (c) were analyzed by RT-qPCR. Data were presented as the mean ± SEM of three independent experiments. ^*∗*^*p* < 0.01 vs. vehicle.

**Figure 4:** EFE inhibits MAPK activation by IL-1*β* in HGFs. Cells were preincubated with the EFE for 1 h and then stimulated with IL-1*β* for 30 min. Using western blotting, the phosphorylated and total MAPK (p38, ERK, and JNK) proteins were quantified (a). Cells were prestimulated with 25 and 50 *μ*g/ml of the EFE for 1 h and then incubated with 0.5 ng/ml of IL-1*β* for 3 h. After nuclear fractionation, western blot analysis was performed to quantify nuclear NF-*κ*B (p65 and p50) and AP-1 (p-c-Jun) subunits (b).

**Figure 5:** EFE inhibits IL-1*β*-induced MAPK/STAT-3 activation in HGFs. Cells were pretreated with 50 *μ*g/ml of the EFE for 1 h and then incubated with IL-1*β* for 3 h. Western blot analysis was performed to confirm the presence of p-STAT-3 and STAT-3 in the nucleus (a). HGFs were pretreated with MAPK inhibitors (p38: SB203580, ERK: PD98059, and JNK: SP600125) for 1 h and then stimulated with IL-1*β* for 3 h. The levels of p-STAT-3 and STAT-3 in nuclear extracts were analyzed by western blotting (b). Cells were transfected with STAT-3 or negative control siRNA for 48 h. STAT-3 protein levels were analyzed by western blot analysis (c). HGFs were transfected for 48 h and then incubated with IL-1*β* for 24 h. Western blot analysis was performed to determine MMP-1 and MMP-3 protein expression (d).

**Table 1:** Primer sequences.

Gene name	Primer sequences
TNF-*α*	Forward: 5′-CTGCTGCACTTTGGAGTGAT-3′
	Reverse: 5′-AGATGATCTGACTGCCTGGG-3′
IL-6	Forward: 5′-TACCCCCAGGAGAAGATTCC-3′
	Reverse: 5′-GCCATCTTTGGAAGGTTCAG-3′
IL-8	Forward: 5′-AGACAGCAGAGCACACAAGC-3′
	Reverse: 5′-ATGGTTCCTTCCGGTGGT-3′
MMP-1	Forward: 5′-AGTGACTGGGAACCGATGCTGA-3′
	Reverse: 5′-CTCTTGGCAAATCTGGCCTGTAA-3′
MMP-3	Forward: 5′-ATTCCATGGAGCCAGGCTTTC-3′
	Reverse: 5′-CATTTGGGTCAA ACTCCAACTGTG-3′
GAPDH	Forward: 5′-ATGGAAATCCCATCACCATCTT-3′
	Reverse: 5′-CGCCCCACTTGATTTTGG-3′

## Data Availability

The data used to support the findings of this study are included within the article.
